# Diagnostic Value of Dynamic Enhanced Magnetic Resonance Imaging Combined with Serum CA15-3, CYFRA21-1, and TFF1 for Breast Cancer

**DOI:** 10.1155/2022/7984591

**Published:** 2022-03-29

**Authors:** Feng Xue, Yu Meng, Jie Jiang

**Affiliations:** ^1^Hepatobiliary Surgery, Qingdao Jiaozhou Central Hospital, Qingdao 266300, Shandong Province, China; ^2^Radiology Department, Jinan Fourth People's Hospital, Jinan 250031, Shandong Province, China; ^3^Radiology Department, Affiliated Hospital of Shandong University of Traditional Chinese Medicine, Jinan 250011, Shandong Province, China

## Abstract

**Objective:**

To explore the diagnostic value of dynamic enhanced magnetic resonance imaging (MRI) combined with serum CA15-3, CYFRA21-1, and TFF1 for breast cancer.

**Methods:**

By means of a retrospective study, 60 breast cancer patients treated in our hospital from January 2018 to December 2020 were selected as the breast cancer group, 60 patients with benign breast lesions were selected as the benign group, and 60 healthy individuals who received physical examination in our hospital in the same period were selected as the control group. All study subjects received dynamic enhanced MRI scan and serological tests, their serum CA15-3 and CYFRA21-1 levels were measured with the electrochemiluminescence instrument and original auxiliary reagent, and the TFF1 level was measured with enzyme-linked immunosorbent assay (ELISA). The MRI performance variation in breast lesion patients was analyzed, the serum CA15-3, CYFRA21-1, and TFF1 levels of study subjects were compared among the three groups, and the efficacy of single diagnosis by dynamic enhanced MRI, CA15-3, CYFRA21-1, or TFF1 as well as combined diagnosis was explored by ROC curves.

**Results:**

Dynamic enhanced MRI showed that malignant lesion had obscure boundary, irregular margin, and heterogeneity after enhancement, and the time-signal intensity curve presented fast-in fast-out; the benign lesion had a clear boundary and smooth margin, 25 cases showed homogeneity after enhancement, and the time-signal intensity curve presented slow-in slow-out; the CA15-3, CYFRA21-1, and TFF1 levels were significantly different among the breast cancer group, benign group, and control group (33.81 ± 12.46 vs 19.02 ± 6.47 vs 9.55 ± 2.64, 4.08 ± 1.41 vs 1.96 ± 1.19 vs 0.99 ± 0.21, 1.39 ± 0.54 vs 1.04 ± 0.26 vs 0.89 ± 0.12, *P* < 0.05); 57 breast cancer patients were diagnosed by a combined examination, with a sensitivity of 95.0%, specificity of 83.3%, positive predictive value of 74.0%, negative predictive value of 97.1%, accuracy rate of 87.2%, and AUC (95%CI) = 0.892 (0.840–0.943), indicating a significantly higher diagnostic value of the combined examination than the single examination by CA15-3, CYFRA21-1, TFF1, or MRI.

**Conclusion:**

Combining dynamic enhanced MRI with serum CA15-3, CYFRA21-1, and TFF1 has good efficacy in diagnosing breast cancer, which can be applied in clinical diagnosis of breast cancer.

## 1. Introduction

Breast cancer is a malignant tumor originating from mammary epithelial cells, and its early manifestations mainly include breast masses and auxiliary lymphadenectasis. With disease progression, distant metastasis of cancer cells may occur, leading to multiple organ lesions, which seriously affect the life health of patients [1]. According to the survey data of the International Agency for Research on Cancer in 2018, the incidence of breast cancer among female malignancies is 24.2% worldwide, with 52.9% occurring in developing countries [2]. China, as the most populous developing country, has a long history of ranking at the top of the globe for a number of breast cancer patients [3]. By 2020, China has 420,000 new cases of breast cancer per year, accounting for 18.6% of the total global cases and ranking first among new cases of malignancies in Chinese women [4, 5]. Although the mortality rate of female breast cancer patients in China is lower than that of lung cancer, colorectal cancer, and gastric cancer, more than 100,000 patients die from breast cancer each year; the number of patients who died from breast cancer in China accounted for 9.6% of the global total in 2008, which still shows an increasing trend [6], so it is extremely important to enhance the secondary prevention of breast cancer before achieving fundamental breakthroughs in the treatment. Early detection and early diagnosis are the core measures of secondary prevention[7], and at present, clinical screening for breast cancer is generally performed by imaging modalities, of which MRI is one of the most widely used methods. MRI has good soft tissue resolution, and dynamic enhanced scanning can further show the lesion morphology and internal blood perfusion, providing physicians with a diagnostic basis. However, comprehensive analysis showed that the diagnostic accuracy of MRI fluctuates greatly, indicating that its diagnostic accuracy is closely related to the experience of physicians [8], so it is difficult to avoid missed diagnosis and erroneous diagnosis in practice and other indicators should be jointly applied to improve the diagnostic accuracy. CA15-3 and CYFRA21-1 are common serological markers, among which CA15-3 is a typical serum marker for breast cancer and is important to guide the diagnosis of breast cancer [9], while CYFRA21-1 has some sensitivity for progressive breast cancer and can assist CA15-3 in diagnosis. In addition to the above typical markers, recent studies have identified TFF1 for playing an important role in the proliferation and apoptosis of cancer cells, which is usually highly expressed in breast cancer tissues, thus representing some value in assessing breast cancer [10]. At the present stage, there are no studies combining dynamic enhanced MRI with CA15-3, CYFRA21-1, and TFF1, but the combination of imaging examination and serologic testing is important for the secondary prevention of breast cancer, so the diagnostic efficacy of combining dynamic enhanced MRI with CA15-3, CYFRA21-1, and TFF1 was explored herein, with the results summarized as follows.

## 2. Materials and Methods

### 2.1. General Data

A total of 60 breast cancer patients treated in our hospital from January 2018 to December 2020 were selected as the breast cancer group, 60 patients with benign breast lesions were selected as the benign group, and 60 healthy individuals who received physical examination in our hospital in the same period were selected as the control group. Patients in the benign group and control group were pathologically diagnosed to exclude malignant lesions and had normal communication skills. All breast cancer patients met the following inclusion criteria: (1) the patients were diagnosed with breast cancer after pathological examination [11]; (2) the patients had not received related treatment before enrollment; (3) the patients had complete clinical data. Exclusion criteria were as follows: (1) the patients could not communicate with others due to hearing disorder, language disorder, and other factors; (2) the patients had distant metastasis of cancer cells; (3) the patients had received treatment measures such as chemotherapy and radio therapy; (4) the patients were complicated or had been complicated with other malignant tumors; (5) the patients were complicated with hematological diseases, autoimmune diseases, and infectious diseases; (6) the patients had dysfunction of important organs; (7) pregnant or lactating women.

All patients in the three groups were females. In the breast cancer group, patients' mean age was (45.37 ± 5.23) years, body mass was (62.12 ± 2.32) kg, and tumor diameter was (17.65 ± 1.23) mm; according to breast cancer TNM staging of Union for International Cancer Control (UICC), there were 4 cases in stage I, 26 cases in stage II, 25 cases in stage III, and 5 cases in stage IV; there were 15 cases with papillary carcinoma, 12 cases with intraductal carcinoma, 23 cases with invasive ductal carcinoma, and 10 cases with carcinoma simplex. In the benign group, patients' mean age was (45.65 ± 5.29) years and body mass was (62.35 ± 2.21) kg; there were 12 cases with breast cyst, 20 cases with fibromatosis of the breast, 5 cases with benign phyllodes tumor of the breast, 15 cases with hyperplasia of mammary glands, and 8 cases with mastitis. In the control group, patients' mean age was (45.38 ± 5.21) years and body mass was (62.41 ± 2.30) kg. No statistical differences in patients' general data including age and body mass among the three groups were observed (*P* > 0.05), presenting value of research.

### 2.2. Moral Consideration

The study met the principles in World Medical Association Declaration of Helsinki (2013)[12], and the study objects signed the informed consent.

### 2.3. Methods

#### 2.3.1. Dynamic Enhanced MRI

The 1.5 T superconducting MRI scanner (MAGNETOM ESSENZA; NMPA Registration Certified no. 20143282054) manufactured by Siemens AG, Germany, was adopted. The study subjects were in the prone position, with the bilateral mammary glands being naturally symmetric and overhanging within the examining hole of a 4-channel phase array surface coil for the breast, and the examinations of cross-sectional T_1_WI sequence, cross-sectional STIR sequence, and sagittal T_2_WI with fat suppression sequence were conducted in turn. Then, dynamic enhanced scanning was performed, the parameters of sagittal plane scanning were TR/TE 4.5 ms/min, FOV 22 cm, matrix 288×160, layer thickness of 3 mm, and flip angle of 15°. 0.2 mL/kg of gadopentetate dimeglumine injection (manufactured by Beijing Beilu Pharmaceutical Co., Ltd.; NMPA approval no. H20013088) was administered to patients at a rate of 3 mL/s, and bolus injection was followed by continuous acquisition for 60 s per phase.

The scanned images were entered into the workstation for image processing, and image evaluation was performed by 3 highly qualified radiologists to observe the boundary, morphology, signal, etc. Of the tumor, after the enhancement, in addition to the routine observation of indicators, the enhancement form of the lesions, the time-signal curve, etc., were observed.

#### 2.3.2. Serologic Tests

*TFF1.* Four ml of fasting venous blood was drawn from the study subjects, let to stand for 20 min, and then centrifuged for 5 min under 3,000 r/min to extract the supernatant, and the TFF1 level was measured with enzyme-linked immunosorbent assay (ELISA) (Beijing Kewei Clinical Diagnostic Reagent Inc.; NMPA approval no. S20060028).

*CA15-3 and CYFRA21-1*. Five ml of fasting venous blood was drawn from the study subjects, let to stand for 20 min, and then centrifuged for 10 min under 3,000 r/min to extract the supernatant, and the CA15-3 and CYFRA21-1 levels were measured with a Switzerland Roche electrochemiluminescence instrument (E602, original auxiliary reagent; NMPA (I) 20113402843).

### 2.4. Determination of Results

1. *MRI*. The results were determined by 3 radiologists through discussion.
2. *Serological Indicators*. CA15-3 ≥ 25 U/ml indicated positive, CYFRA21-1 ≥ 3.5 ng/mL indicated positive, and TFF1 S/*N* value (S: specimen A value; N: negative control A value) ≥ 2.1 indicated positive. When combining the three serological indicators and MRI in diagnosis, if any result was positive, it was determined as positive, and if four results were negative, it was determined as negative.
3. *Diagnostic Efficacy*. ① Sensitivity: the number of true positive cases/(the number of true positive cases + the number of false negative cases) ∗ 100%; ② specificity: the number of true negative cases/(the number of true negative cases + the number of false positive cases) ∗ 100%; ③ positive predictive value (PPV): the number of true positive cases/(the number of true positive cases + the number of false positive cases); ④ negative predictive value (NPV): the number of true negative cases/(the number of false negative cases + the number of true negative cases).

### 2.5. Statistical Processing

In this study, the data processing software was SPSS20.0, the picture drawing software was GraphPad Prism 7 (GraphPad Software, San Diego, USA), the items included were enumeration data and measurement data, the methods used were X^2^ test and *t*-test, and differences were considered statistically significant at *P* < 0.05.

## 3. Results

### 3.1. Analysis of Patients' MRI, Performance

MRI of the breast cancer group showed an obscure boundary and irregular margin. On routine MRI, 40 cases showed long *T*_1_ and long *T*_2_, 5 cases showed short *T*_1_ and long *T*_2_, and 58 cases showed hyperintensity on T_2_WI and in 42 cases, early enhancement was seen on contrast-enhanced scans and the enhancement was not uniform. In terms of the time-signal intensity curves, there were 3 cases of the inflow type, 15 cases of the plateau type, and 42 cases of the outflow type.

MRI of the benign group showed a clear boundary and smooth margin, in a quasi-circular, circular, or leaf shape, and hyperintensity, isointensity, or hypointensity on T_1_WI. No enhancement was seen on contrast-enhanced scans of 35 cases, and in 25 cases, the enhancement was uniform. In terms of the time-signal intensity curves, there were 45 cases of the inflow type, 13 cases of the plateau type, and 2 cases of the outflow type.

### 3.2. Comparison of Study Subjects' Serological Indicators

The CA15-3, CYFRA21-1, and TFF1 levels were significantly higher in the breast cancer group than in the benign group and control group (*P* < 0.05) (Figure 1).

The CA15-3, CYFRA21-1, and TFF1 levels were significantly different among the breast cancer group, benign group, and control group (33.81 ± 12.46 vs 19.02 ± 6.47 vs 9.55 ± 2.64, 4.08 ± 1.41 vs 1.96 ± 1.19 vs 0.99 ± 0.21, 1.39 ± 0.54 vs 1.04 ± 0.26 vs 0.89 ± 0.12, *P* < 0.05).

### 3.3. Diagnostic Results of Different Diagnosis Modalities

For results of single diagnosis by CA15-3, CYFRA21-1, TFF1, or MRI and of combined examination, see Table 1.

### 3.4. Diagnostic Efficacy of Different Diagnosis Modalities

For the diagnosis efficacy of CA15-3, CYFRA21-1, TFF1, and MRI, see Table 2. The combined examination had a sensitivity of 95.0%, specificity of 83.3%, PPV of 74.0%, NPV of 97.1%, accuracy rate of 87.2%, and AUC (95%CI) = 0.892 (0.840–0.943), indicating a diagnostic efficacy significantly higher than single examination by CA15-3, CYFRA21-1, TFF1, or MRI (Figure 2).

## 4. Discussion

Breast cancer, a malignancy resulting from uncontrolled proliferation of mammary epithelial cells, occurs more often in women and less frequently in men[13]. The mortality rate of breast cancer has gradually declined worldwide with increasing medical levels in recent years [14], but the incidence and mortality rates in China have not reduced in synchrony and related data show that in 2020, China had 420,000 breast cancer patients and 120,000 patients died from the disease, which are significantly increasing compared to the data in 2018, indicating that the social and economic transition in China causes constant changes in risk factors for breast cancer [15, 16]. Increasing emphasis on risk factors is the primary prevention of breast cancer, and enhancing the ability of early screening and early diagnosis is the secondary prevention measure [17, 18]. Primary prevention aims to reduce the incidence of breast cancer, whereas secondary prevention aims to prevent further deterioration of the initial breast cancer, so that patients will not lose the optimal timing of treatment, and therefore, secondary prevention is essential to improve patients' survival. Secondary prevention measures for breast cancer are to define the nature of the lesion based on the level of serum tumor markers in patients, comprehensive assessment of imaging examinations, and surveillance for the occurrence of breast cancer, and, if necessary, pathological biopsy [19]. Since the pathological biopsy is invasive and there is a negative effect on the normal tissue of the body, it is not recommended when it is not necessary and obtaining pathology samples from all patients in the clinic is not practical. Compared with pathological biopsy, imaging examination and serological tests are more convenient, which can meet the needs of breast cancer screening in China with a large population base according to the local condition. MRI is the most commonly used imaging modality for breast cancer in clinics, which has no ionizing radiation and therefore will not cause radiation damage and has a good rate of soft tissue resolution, and after injecting contrast agents for dynamic enhanced scanning, the blood flow perfusion inside the lesion tissue can be clearly shown, which helps physicians in making decisions from the degree of lesion enhancement, morphological characteristics, etc. [20, 21]. The study results showed that the dynamic enhanced MRI image of breast cancer lesions had an obscure boundary and irregular margin and was not uniform after enhancement, which was due to the presence of a large number of neovessels within the lesions, so enhancement was obvious after contrast-enhanced scanning in most lesions; in addition, with high microvessel density and vascular permeability of lesion, the time-signal intensity curve showed fast-in fast-out. Compared with breast cancer lesion, a typical benign breast lesion had a clear boundary and smooth margin, and among 60 patients with benign breast lesions in the study, the time-signal intensity curve in 25 cases showed slow-in slow-out, which was significantly different from the breast cancer lesion. It should be noted that some benign lesions may still be misdiagnosed as malignant lesions, so MRI is best complemented by serological tests to increase the detection rate.

Currently, CA15-3 is one of the most common serum markers of breast cancer, which is a variant of the epithelial surface glycoprotein of breast cells, was first found on the breast cancer cell pellicle, and exhibits a high expression status in breast cancer tissue, so it can be used to determine the condition of breast cancer lesions[22]. The diagnostic efficacy of CA15-3 for breast cancer has been recognized by the academic community, and compared with CYFRA21-1, it belongs to the more novel breast cancer diagnostic markers. Although it was confirmed to have high sensitivity in some studies, scholars Bayo J et al. found that CYFRA21-1 only has a good diagnostic value for intermediate, advanced, and recurrent breast cancer [23], and its sensitivity for early breast cancer is extremely low. This study found a diagnostic sensitivity of 60.0% for CA15-3 and 56.7% for CYFRA21-1, presumably related to the patient sample selected herein. In addition to CA15-3 and CYFRA21-1, TFF1 is also closely related to breast cancer. TFF1 belongs to the trefoil factor family, which plays an important role in various types of physiological activities in the body; normally, it is less expressed in the mammary gland, and in case of overexpression, it will cause female estrogen imbalance and at the same time increase cyclin D1 and accelerate the proliferation of breast tissue cells [24] and eventually induce breast cancer. Latest studies showed that TFF1 can be used in the diagnosis and efficacy evaluation of breast cancer [25], and this study found that the sensitivity of TFF1 was 66.7%, which could be up to 95.0% when combining with CA15-3, CYFRA21-1, and MRI; its diagnostic accuracy rate was 87.2% and AUC (95%CI) = 0.892 (0.840–0.943), indicating that the diagnostic efficacy of combined diagnosis was significantly higher than that of single examination by CA15-3, CYFRA21-1, TFF1, or MRI.

In conclusion, breast cancer is a relatively common malignancy in the clinical field and increasing the detection rate of this disease is beneficial for reducing the medical burden of breast cancer in China. The study found that combining dynamic enhanced MRI with serum CA15-3, CYFRA21-1, and TFF1 has a good efficacy in diagnosing breast cancer, which can be applied in the clinical diagnosis of breast cancer.

## Figures and Tables

**Figure 1:** Comparison of study subjects' serological indicators (*x* ± *s*). Note: (a) the CA15-3 level; (b) the CYFRA21-1 level; and (c) the TFF1 level.

**Figure 2:** Analysis of diagnostic efficacy of different diagnosis modalities by ROC curves.

**Table 1:** Diagnostic results of different diagnosis modalities.

Pathologic findings	CA15-3+ -		CYFRA21-1+ -		TFF1+ -		MRI + -		Combined examination + −		Total
+	36	24	34	26	40	20	35	25	57	3	60
-	18	102	16	104	19	101	16	104	20	100	120
Total	54	126	50	130	59	121	51	129	77	103	180

**Table 2:** Diagnostic efficacy of different diagnosis modalities.

Group	Sensitivity (%)	Specificity (%)	PPV (%)	NPV (%)	Accuracy rate (%)
CA15-3	60.0 (36/60)	85.0 (102/120)	66.7 (36/54)	81.0 (102/126)	76.7 (138/180)
CYFRA21-1	56.7 (34/60)	86.7 (104/120)	68.0 (34/50)	80.0 (104/130)	76.7 (138/180)
TFF1	66.7 (40/60)	84.2 (101/120)	67.8 (40/59)	83.5 (101/121)	78.3 (141/180)
MRI	58.3 (35/60)	86.7 (104/120)	68.6 (35/51)	80.6 (104/129)	77.2 (139/180)
Combined examination	95.0 (57/60)	83.3 (100/120)	74.0 (57/77)	97.1 (100/103)	87.2 (157/180)

## Data Availability

The data used to support the findings of this study are available on reasonable request from the corresponding author.
